The article "Study on Spontaneous Combustion “Three Zones” of the Distribution Law and Integrated Fire Prevention Technology in Mined-Out Area of Lingquan Mine" was published in 2022. Journal: Comput Intell Neurosci.

# Study on Spontaneous Combustion “Three Zones” of the Distribution Law and Integrated Fire Prevention Technology in Mined-Out Area of Lingquan Mine

**DOI:** 10.1155/2022/4005954

**Published:** 2022-04-18

**Authors:** Linjie Liu, Zhuo Shen, Jian Chen, Baoshan Jia, Guorui Su, Rongzheng Liu

**Affiliations:** ^1^College of Safety Science and Engineering, Liaoning Technical University, Fuxin, Liaoning 123000, China; ^2^Key Laboratory of Mine Thermodynamic Disasters and Control of Ministry of Education, Liaoning Technical University, Fuxin, Liaoning 123000, China; ^3^Information Institute of the Ministry of Emergency Management of PRC, Beijing, China

## Abstract

To determine the risk range of remaining coal in the goaf of the higher slice on the seventh mining and fifth face of Lingquan Mine, the beam tube monitoring system was adopted to supervise the temperature and gas content changes in the goaf during the normal mining period of the working face. As per the principle of dividing spontaneous combustion “three zones” (SCTZ), numerical simulation of the distribution of SCTZ in the goaf of the work face was performed. The O_2_ content and index gas in the goaf were measured and analyzed, and combined with the in-situ measurement outcomes, the distribution of SCTZ in the goaf was determined through the FLUENT numerical modeling program. The outcomes show that the distribution pattern of SCTZ in the goaf of fully mechanized mining face is: the heat dissipation zone is 0–41 m, the oxidation zone is 41–97 m, the suffocation zone is more than 97 m away from the work face, and the increment of temperature is 0.7/°C. Based on the judgement result of SCTZ, the minimum recovery rate of work face is above 3.7 m/d. The use of new polymer materials validly solves the problem of excessive CO in the return air corner of the goaf and prevents self-ignition accidents in the goaf.

## 1. Preface

Spontaneous ignition of residual coal is one of the factors that threaten the safety of mine production and cause major hazards. According to statistics, among the 658 key coal mines in the country, 55.8% of them have a tendency to spontaneous combustion, and 52% of them have the shortest self-ignition period that less than 3 months[1]. O_2_ concentration is one of the necessary conditions for coal self-ignition. Considering factors such as accuracy, feasibility, and efficiency, we often use O_2_ concentration as a monitoring indicator in practice. We usually divide SCTZ in the mined-out area into heat dissipation, oxidation and suffocation zones according to air leakage, O_2_ concentration, and temperature [2](Table 1). This paper has taken the higher slice working face on the seventh mining and fifth face of Lingquan Mine as the object of study. Adopting the beam tube monitoring system theory, and referring to the results of field measurement and numerical modeling, the distributing range of the SCTZ in the goaf was determined. On the foundation of the latest self-ignition period analysis report and the minimum recovery rate of the work face, a scientific theoretical guidance was provided to prevent the self-ignition of the residual coal in the goaf of Lingquan Mine.

The article "Study on Spontaneous Combustion “Three Zones” of the Distribution Law and Integrated Fire Prevention Technology in Mined-Out Area of Lingquan Mine" was published in 2022. Journal: Comput Intell Neurosci.

## 2. Overview of the Mine

Lingquan Mine is affiliated to the Dalai Nur mining area, Manzhouli City, Hulunbuir City, Inner Mongolia Autonomous Region. It is 7.4 km long in the north-south direction, 4.2 km wide in the east-west slope, and has a total area of 31.1 km^2^. The reserve resources within the mine are 43.723 million tons, the mineable coal is lignite, and the mineable reserves are 23.729 million tons.

In 2021, the spontaneous combustion tendency of the II_3_ coal seam (sampling location: higher slice on the seventh mining and fifth face) was graded and the spontaneous combustion period was tested and analyzed. The outcomes indicated that the self-ignition tendency grade of coal seam was Class II, the shortest self-ignition period was 39 days, the maximum absolute gas emission rate registered 0.52 m^3^/min, the relative gas emission rate registered 0.67 m^3^/*t*, the oxygen absorption content of coal is 0.54 cm^3^/g, the thickness of coal bed is 18.5 m, the coal bed inclination was 1°C-5°C, and the equivalent specific heat capacity of the sample is 2.381 J/g·k. It belongs to the full mechanization mining face in ultrathick coal bed, with low gas and easy to self-ignition.

## 3. Measurement and Analysis of the SCTZ in the Goaf

### 3.1. Analysis of “Three Zones”

According to the pressure of the collapsed rock mass, the goaf is usually divided into the original rock stress zone, the stress concentrated area the low stress area, the stress recovery area and the recompaction area (respectively, represented by 1.2. 3.4. 5 in Figure 1). The “caving zone” in the goaf forms zone I, zone II, and zone III (as shown in Figure 1), which are natural accumulation zone, broken accumulation zone, and re-compaction zone respectively [3–6]. Zone I is the closest to the work face. The coal or rock mass in the goaf is in a loose state, the amount of air leakage is large and the speed is fast, and the heat produced by coal oxidation dissipates quickly, which is similar to the cooling zone in the SCTZ. In zone II, the coal or rock mass in the goaf seems dense, but there are still air leakage channels, so substantial heat generated by coal oxidation is dissipated. However, the heat of the coal is accumulated, causing it to heat up, which is similar to the oxidation zone in the SCTZ. In zone III, the coal or rock mass in the goaf is crushed and compacted under the pressure of the overlying rock. The porosity is small, the O_2_ content of the remaining coal becomes low, and the coal is almost not oxidized, which is similar to the suffocation zone in the SCTZ [4, 5].

The article "Study on Spontaneous Combustion “Three Zones” of the Distribution Law and Integrated Fire Prevention Technology in Mined-Out Area of Lingquan Mine" was published in 2022. Journal: Comput Intell Neurosci.

### 3.2. Layout of Beam Tubes in the Goaf

To determine the distribution range of SCTZ, the method of pre-embedded beam tubes and temperature sensors was adopted to observe the gas composition, concentration and temperature in the goaf [4, 5]. As per the reality of the work face, three measuring points (1^#^, 2^#^, 3^#^) were laid at the back chute, with a distance of 30 m between each measuring point, and one measuring point was laid for each of the inlet and return air corners (5^#^, 4^#^), with a distance of 230 m. Each measuring point was composed of a beam tube and a temperature probe. Two measuring points (upper tunnel: 8^#^, 9^#^, lower tunnel: 6^#^, 7^#^) were laid symmetrically along the wall in the two tunnels of inlet and return air. Each measuring point had only one beam tube, and the distance between the sampling head of each beam tube was 30 m (as shown in Figure 2). Based on the current mining technology and the oxidation characteristics of the remaining coal in the mined-out area, the beam tube extraction device was placed in the well. At each measuring point, researchers used a combination of manual and electric gas extraction methods to bring the collected airbags back to the ground. Based on gas chromatography research and analysis (as shown in Figure 3), the changes in the content of O_2_ and other gas in the mining process in the goaf were summarized.

As the working face advance, gas sampling and temperature measurement were performed at nine measuring points regularly to obtain real-time indicators of temperature and gas concentration for different advance distances in the goaf. As per the theory of self-ignition of residual coal, and referring to the change law of the O_2_ content and temperature in the mined-out area with the depth of the goaf, the distribution range of the SCTZ in the goaf was determined. Due to the collapsed rocks and pondings in the mined-out area, the roof fall in the mined-out area would cause blockage of the beam tube and the probe. To effectively avoid this phenomenon, the following measures were specially formulated (as shown in Figure 4): ① A tee pipe with a length of 1 m was welded at each measuring point, three on the inlet side and return side, perpendicular to the 2-inch steel pipe; ② ten to twenty air-permeable small holes with a diameter of 8 mm were drilled around the front end of the casing at 0.50 m, which could not only realize the function of gas extraction, but also temperature measurement; ③ to prevent gas from being extracted from the casing, foaming agent was used to block the 2-inch steel pipe near the tee.

The article "Study on Spontaneous Combustion “Three Zones” of the Distribution Law and Integrated Fire Prevention Technology in Mined-Out Area of Lingquan Mine" was published in 2022. Journal: Comput Intell Neurosci.

### 3.3. Analysis of Measured Data

#### 3.3.1. Analysis of O_2_ Concentration Data at Measuring Points in the Goaf

Based on the data collected by these measuring points, the changing curve of oxygen concentration of each measuring point with the advancing distance of the work face is presented in the figures below. From the measurement results, the volumetric fraction of O_2_ at the air inlet corner is higher, and the volumetric fraction at the return airflow corner is lower, which conforms to the airflow law in the mined-out area. The oxygen concentration changes of 1^#^∼3^#^ measuring points at the back chute are presented by Figure 5, With the work face advance to 35 meters, the oxygen mass fraction of measuring point 3^#^ is lower than 18%. Measuring point 3^#^ is the first to enter the oxidation zone, while 1^#^ and 2^#^ enter the oxidation zone at 41.5 m and 40.8 m, respectively. The coal is further compacted, and this goaf is remining and has the characteristics of extrathick coal seams. Therefore, when the advancing distance of the work face reaches 79.5 m, the O_2_ content of measuring point 3^#^ drops below 8%, indicating that it has entered the suffocation zone (as shown in Table 2).

According to the measured data and the above-mentioned two-dimensional diagrams, nine measurement points were drawn with the increase of buried depth and the three-dimensional diagram of the O_2_ content distribution of each measuring point was drawn with Origin. Under ideal conditions, this picture can clearly reflect the different oxygen content changes at the air inlet side, return airflow side, air inlet corner, return air corner, and back chute in the mined-out area, for the purpose of determining the distribution of the “three zones”.. (as shown in Figure 6).

#### 3.3.2. Analysis of Temperature Data in the Goaf

If there is oxidation heating in the goaf, the temperature monitoring can clearly measure the change law of stope temperature, which can be used as an index to divide the SCTZ in the goaf [7]. However, if there is no oxidation heating in the goaf, the temperature can only be used as a reference factor. As the working face advances, the temperature change of the measuring point in the goaf is shown in Figure 7. For the measuring point 5^#^ at the air inlet corner, when the burial depth is from 40 m to 73 m, the temperature rises from 19.80°C to the highest point 23.4°C, and then the temperature is in a fluctuating state. For the measuring point 4^#^ at the return air corner, when the burial depth is from 25 m to 60 m, the temperature rises from 16.50°C to the highest point 20.32°C, and then the temperature also fluctuates. In summary, the temperature at the measurement point in the goaf shows a certain regularity, with an increment of 0.7°C/d, so it can be used as the basis for dividing the cooling zone and the oxidation zone.

The article "Study on Spontaneous Combustion “Three Zones” of the Distribution Law and Integrated Fire Prevention Technology in Mined-Out Area of Lingquan Mine" was published in 2022. Journal: Comput Intell Neurosci.

## 4. Numerical Simulation

### 4.1. Parameter Setting

Adopting efficient FLUENT software, the O_2_ concentration in the goaf was numerically simulated. Based on the structure-related principles of the mass, momentum, and composition of the gas flowing in porous media, in order to meet the simulation requirements and referring to the law of conservation of momentum, the following equations were proposed [8, 9]:

(1) $$\begin{array}{c} \frac{\partial \rho }{\partial t}+\nabla \left(\rho v\right)=H_{\text{p}}, \end{array}$$

where *ρ* is density, *v* is speed, t is time, and *H*_*p*_ is source item.

(2) $$\begin{array}{c} \frac{\partial }{\partial t}\left(\rho {\text{y}}_{i}\right)+\frac{\partial }{\partial x_{j}}\left(\rho y_{i}y_{j}\right)=-\frac{\partial p}{\partial x_{i}}+\frac{\partial q_{ij}}{\partial x_{j}}+\rho g_{i}+H_{i}, \end{array}$$

where *H*_*i*_ is the momentum loss source item in *i* direction, *g*_*i*_ is the gravity volume in *i* direction, P is pressure, *y*_*i*_*y*_*j*_ is the velocity component in *i* direction and *j* direction, *x*_*i*_*x*_*j*_ is the *i* direction and *j* direction in three-dimensional space, and *q*_*ij*_ is the viscous stress component.

(3) $$\begin{array}{c} H_{i}=\sum_{j=1}^{5}B_{ij}uv_{j}+\sum_{j=1}^{5}F_{ij}\frac{1}{2}\rho \left|v_{j}\right|v_{j}, \end{array}$$

where *u* is viscosity, *B*_*ij*_*F*_*ij*_ is the corresponding prescribed coefficient matrix, and *v*_*j*_ is the velocity component.

(4) $$\begin{array}{c} \frac{\partial \left(\rho F_{S}\right)}{\partial t}+\mathrm{div}\left(\rho uF_{S}\right)=\mathrm{div}\left\{B_{S}\mathrm{grad}\left(\rho F_{S}\right)\right\}+S_{S}, \end{array}$$

where *F*_*S*_ is the volume concentration of component S, *B*_*s*_ is the volume fraction of component S, and *S*_*S*_ is the mass of component S in the goaf.

(5) $$\begin{array}{c} \frac{\partial \left(\rho T\right)}{\partial t}+\mathrm{div}\left(\rho uT\right)=\mathrm{div}\left(\frac{k}{F_{\text{p}}}\mathrm{grad}T\right)+H_{\text{T}}, \end{array}$$

where *F*_p_ is the specific heat capacity, *T* is the thermodynamic temperature, *k* is the thermal conductivity of the goaf, and *H*_T_ is the energy source item.

The article "Study on Spontaneous Combustion “Three Zones” of the Distribution Law and Integrated Fire Prevention Technology in Mined-Out Area of Lingquan Mine" was published in 2022. Journal: Comput Intell Neurosci.

The above equations are based on the gas flow in the goaf, and the necessary basic conservation equations are established. After further setting the original conditions and boundary conditions [9], the key parameters and UDF custom functions are imported into the FLUENT solver for solution, then the distribution law of oxygen concentration in the goaf can be obtained.

Based on the related theories of the goaf seepage and diffusion mathematical model [10], a numerical model of the higher slice working face on the seventh mining and fifth face was established. The size of the goaf is 400 m × 220 m × 60 m; the size of the full mechanization mining face is 10 m × 220 m × 4 m; the size of the inlet and outlet tunnel of the full mechanization mining face is 20 m × 4 m × 3.5 m. The model is divided into 26189 grids and 130413 nodes (as shown in Figure 8). U-shaped ventilation is adopted in the model, starting with the air inlet tunnel and coming out of the return air tunnel, each with a width of 4 m, and an air volume distribution of 1000 m^3^/min. The mining operation of the working face is continued, so does the analysis of the seepage field in the goaf.

### 4.2. Numerical Simulation Results and Comparative Analysis with Measurement Results

The simulation results of the FLUENT software were optimized by Tecplot software, and the O_2_ content distribution map of the goaf was obtained, which could provide more accurate theoretical reference values for the division of “three zones”.

The static pressure difference between the air inlet tunnel and the return airflow tunnel of the higher slice working face on the seventh mining and fifth faces was 105 Pa. Under ventilation conditions, the internal pressure distribution in the mined-out area was arc-shaped due to the air intake. The pressure gradually decreases from the air inlet side to the return airflow side. The air leak velocity in the middle of the mined-out area was lower than that on the inlet side and return airflow side. It could be obviously observed from the figure that the O_2_ content on the inlet side was significantly lower in contrast to that on the return airflow side [11], the O_2_ content on the inlet side was 22.1%, and the return airflow side was 7.6%. In addition, it could be determined by simulation that when the air air leak velocity was over 0.004 m/s, the goaf was in the heat dissipation zone; when the air leak velocity was within the range of 0.004～0.0017 m/s, the goaf was in the oxidation zone; and when the air leak velocity was below 0.0017 m/s, the goaf was in the suffocation zone (Figures 9 and 10). The results were consistent with the above “three-zone” distribution judgement, which verified the accuracy of the research results (Table 3).

The article "Study on Spontaneous Combustion “Three Zones” of the Distribution Law and Integrated Fire Prevention Technology in Mined-Out Area of Lingquan Mine" was published in 2022. Journal: Comput Intell Neurosci.

### 4.3. Calculation of Minimum Recovery Rate

If spontaneous combustion occurs in the residual coal in the mined-out area of a full mechanization mining face, the residual coal must be thick enough and the oxidation time reaches the shortest spontaneous combustion period. Both conditions must be met at the same time to oxidize the residual coal [12].

(6) $$\begin{array}{c} T(\rangle T_{\text{min}},\\ V(\rangle V_{\min}=\frac{2\left(L_{Z}+L_{b}\right)}{{\text{T}}_{\min}}, \end{array}$$

where *T*_min_ is the shortest spontaneous combustion period, *V*_min_ is the minimum recovery rate that leads to self-ignition of the remaining coal, *L*_*Z*_ is the width of the self-ignition zone, and *L*_*b*_ is the cooling zone width, 2-the safety factor [13].

The average cooling zone length and the spontaneous combustion zone of the fully mechanized mining face was 72.6 m, and the shortest self-ignition period of the II_3_ coal bed is 39 d. Therefore, according to the above equations, the minimum recovery rate of the higher slice work face on the seventh mining and fifth face was 3.7 m/d.

### 4.4. Onsite Fire-fighting Applications

It mainly adopts comprehensive fire-fighting measures such as CO_2_ and nitrogen injection, chemical inhibitor spraying, and postmining water and sand filling and sealing [14]. A bunker was set up near the higher slice working face on the seventh mining and fifth face, and the method of reducing the air supply and blocking the air leakage channel was adopted to extinguish the fire. The volume of the Sanxie bunker is 350 m^3^, the volume of the reservoir is 200 m^3^, and the water supply source is the drainage of the 270 South Pumping Station. It is responsible for the filling of the old Sanxie area and the seventh mining area underground. There are three sets of nitrogen injection fire-fighting systems in the mine, among them, two DM-1000 membrane separation nitrogen generators are installed in the nitrogen injection machine room of the main lane on the right track of the seventh mining area, serving for fire extinguishment and fire fighting in the seventh mining area. The two sets of nitrogen injection machines are of the same model. A mobile inhibitor pump is installed in the train switch area of the upper tunnel on the full mechanization mining face and equipped with a liquid storage tank. The inhibitor pump sends the inhibitor liquid to the coal mining face and the inlet and return air corners through the Φ19 mm pipeline. A valve and spray gun are installed at the end, and the angle and direction of them can be adjusted in time according to the change of spraying inhibitor position.

The article "Study on Spontaneous Combustion “Three Zones” of the Distribution Law and Integrated Fire Prevention Technology in Mined-Out Area of Lingquan Mine" was published in 2022. Journal: Comput Intell Neurosci.

According to the simulation results of the SCTZ range in the goaf, when the air supply is 1,000 m^3^/min, the suffocation zone is 75 m away from the inlet side of the work face, and the CO in the return airflow corner is excessive, which indicates that there is serious air leak in the mined-out area. The main feature of air leak in the goaf is that the air enters from the inlet side and then flows out near the return airflow side, therefore, in order to stop the leakage in the goaf, it is necessary to seal the inlet and return airflow side, the air inlet tunnel and the connection tunnel [15]. The sealing measures adopted are as follows: at the corner of the return airway, a mixture of sodium polyacrylate, polyacrylamide, additives and water in a ratio of 3 : 1:2 : 3 is used to make a new polymer colloid material for sealing, and the connection tunnel is sealed at the same time. Then the high-strength composite foaming plugging material slurry is filled around the colloid and the connection tunnel, so that the collapsed rock and the plugging material form a wall to block the air leak in the mined-out area, thereby preventing the self-ignition of the floating coal.

In view of the spontaneous combustion circumstance of the higher slice work face on the seventh mining and fifth face, the colloid is used to quickly seal the leakage at the corners of the inlet and return air tunnels in the goaf. This material has advantages such as good expansion ability, low dosage, antistatic, and cost saving. It can make the filling of connection tunnels, upper and lower corners more closed, which effectively prevents air leak in the mined-out area and shortens the oxidation zone width. To prevent air leak in the connection tunnel behind the goaf after the work face is advanced, a new type of polymer material plugging system is further adopted. The colloid is used as the framework and filled with high-strength foam concrete to form a leak-proof wall, which can not only stop leakage, but also strengthen coal pillars to reduce the generation of broken coal. Therefore, the CO content in the return airflow corner of the work face and within the working face tends to be stable.

## 5. Conclusion

1. The Fluent numerical modeling program was adopted to simulate the SCTZ range in the goaf under the actual working conditions of the higher slice working face on the seventh mining and fifth face of Lingquan Mine, and the simulation outcomes coincided with the measured outcomes.
2. Through the measurement and analysis of the temperature in the goaf, it can be seen that during the measurement, the temperature at each point was not high, indicating that there was no spontaneous combustion in the mined-out area during the test, and the high temperature zone in the goaf appeared within 45 ∼ 70 m from the workface.
3. Under the condition that the air distribution rate is 1,000 m^3^/min, the maximum oxidation zone width on the back chute side is 56 m, and the narrowest width of the air inlet tunnel is 29 m. The distribution range of the “three zones” in the mined-out area of the fully mechanized mining face is: the heat dissipation zone is 0∼41 m, and the wind speed is above 0.004 m/s; the oxidation zone is 41∼97 m, and the wind speed ranges from 0.004 to 0.0017 m/s; the distance between the suffocation zone and the work face is greater than 97 m, and the wind speed is less than 0.0017 m/s. The increment of temperature is 0.7/°C, and the minimal safe advancing velocity of the work face is 3.7 m/d.
4. Based on the spontaneous combustion law of Type II spontaneous combustion coal seams, in view of the actual mining conditions of the higher slice working face on the seventh mining and fifth face, some fire-fighting pretreatments have been adopted, such as installing isolation walls and spraying sealing materials at the end of track transportation road and the end of the belt transportation road at the stop mining face, and constructing fire-fighting boreholes and injecting colloids between the two ends and the frame. It solves the problem of excessive CO content at the return air corner of the work face, and realizes safe mining on the work face. The width of the oxidation zone is obviously reduced after sealing under the same air volume.

The article "Study on Spontaneous Combustion “Three Zones” of the Distribution Law and Integrated Fire Prevention Technology in Mined-Out Area of Lingquan Mine" was published in 2022. Journal: Comput Intell Neurosci.

## Figures and Tables

**Figure 1:** Horizontal distribution of overlying rock failure in the goaf.

**Figure 2:** Schematic diagram of measuring point layout in the goaf.

**Figure 3:** Ground beam tube analysis device.

**Figure 4:** Structure diagram of gas extraction device.

**Figure 5:** Oxygen concentration change curve of each measuring point in goaf.

**Figure 6:** Three-dimensional diagram of oxygen concentration changing with burial depth at each measuring point in the goaf.

**Figure 7:** Contrast curve of temperature changes of inlet and return air corners in the goaf.

**Figure 8:** Physical model establishment and meshing.

**Figure 9:** Simulated diagram of oxygen distribution in the goaf.

**Figure 10:** Simulation of air leak velocity in the mined-out area.

**Table 1:** Spontaneous combustion “three zones” division.

Index	Basis	Heat dissipation zone	Oxidation zone	Suffocation zone
O_2_ content	O_2_ concentration in the goaf (%)	＞19	9–19	＜9
Speed of air leakage	Speed of air leak in the goaf (m/s)	＞0.0045	0.0016–0.0045	＜0.0016
Temperature	Temperature in the goaf (°C/d)	Take the 1°C/d increasing gradient as the boundary condition between oxidation zone and heat dissipation zone (for reference only)		

The article "Study on Spontaneous Combustion “Three Zones” of the Distribution Law and Integrated Fire Prevention Technology in Mined-Out Area of Lingquan Mine" was published in 2022. Journal: Comput Intell Neurosci.

**Table 2:** Range of measuring points for “three zones.”

Measuring point	Heat dissipation zone	Oxidation zone	Suffocation zone
1^#^	0–41.5 (m)	41.5–95.6 (m)	＞95.6 (m)
2^#^	0–40.8 (m)	40.8–86.0 (m)	＞86.0 (m)
3^#^	0–35.0 (m)	35.0–79.6 (m)	＞79.6 (m)
4^#^	0–25.0 (m)	25.0–60.0 (m)	＞60.0 (m)
5^#^	0–43.0 (m)	43.0–72.0 (m)	＞72.0 (m)

**Table 3:** The distribution law of “three zones” combined with measurement and simulation in the goaf.

Position	Heat dissipation zone/m	Oxidation zone/m	Suffocation zone/m	Maximum width of oxidation zone/m
Return air side	＜25	25–62	＞62	37
Middle	＜40	40–96	＞96	56
Air inlet side	＜46	46–75	＞75	29

## Data Availability

The data that support the findings of this study are available from the corresponding author upon reasonable request.
